The article "The predictive value of BTG1 for the response of newly diagnosed acute myeloid leukemia to decitabine" was retracted in 2024. Reasons: no approval from the institution; concerns about the data.

# The predictive value of BTG1 for the response of newly diagnosed acute myeloid leukemia to decitabine

**DOI:** 10.1186/s13148-024-01627-9

**Published:** 2024-01-22

**Authors:** Yi Li, Xia Mao, Mengyuan Li, Li Li, Xiwen Tong, Lifang Huang

**Affiliations:** 1 Renmin Hospital of Wuhan University, Wuhan, China; 2 Department of Hematology, Tongji Hospital, Tongji Medical College, Huazhong University of Science and Technology, 1095 Jie-fang Avenue, Wuhan, 430030 Hubei China; 3 Xinqiao Hospital of Army Medical University, Chongqing, China

**Keywords:** Acute myeloid leukemia, Decitabine, BTG1, Methylation, Response prediction

## Abstract

**Background:**

Decitabine has been widely used to treat acute myeloid leukemia (AML); however as AML is a heterogeneous disease, not all patients benefit from decitabine. This study aimed to identify markers for predicting the response to decitabine.

**Methods:**

An intersection of in vitro experiments and bioinformatics was performed using a combination of epigenetic and transcriptomic analysis. A tumor-suppressor gene associated with methylation and the response to decitabine was screened. Then the sensitivity and specificity of this marker in predicting the response to decitabine was confirmed in 54 samples from newly diagnosed AML patients treated with decitabine plus IA regimen in a clinical trial (ChiCTR2000037928).

**Results:**

In vitro experiments showed that decitabine caused hypomethylation and upregulation of BTG1, while downregulation of BTG1 attenuated the inhibitory effect of decitabine. In newly diagnosed AML patients who received decitabine plus IA regimen, the predictive value of BTG1 to predict complete remission (CR) was assigned with a sensitivity of 86.7% and a specificity of 100.0% when BTG1 expression was < 0.292 (determined using real-time quantitative PCR), with area under the curve (AUC) = 0.933,* P* = 0.021. The predictive value of BTG1 to predict measurable residual disease (MRD) negativity was assigned with a sensitivity of 100.0% and a specificity of 80.0% when BTG1 expression was < 0.292 (AUC = 0.892, *P* = 0.012). Patients were divided into low and high BTG1 expression groups according to a cutoff of 0.292, and the CR rate of the low-expression group was significantly higher than that of the high-expression group (97.5% vs. 50%,* P* < 0.001).

**Conclusions:**

Low expression of BTG1 was associated with CR and MRD negativity in newly diagnosed AML patients treated with a decitabine-containing regimen, suggesting that BTG1 is a potential marker for predicting the response to decitabine in newly diagnosed AML.

*Clinical trial registration*: ChiCTR2000037928.

**Supplementary Information:**

The online version contains supplementary material available at 10.1186/s13148-024-01627-9.

The article "The predictive value of BTG1 for the response of newly diagnosed acute myeloid leukemia to decitabine" was retracted in 2024. Reasons: no approval from the institution; concerns about the data.

## Introduction

Hypomethylating agents have shown promising efficacy in treating acute myeloid leukemia (AML); however, the complete remission (CR) rate was shown to range from 50.0 to 70.0% in patients treated with decitabine-containing chemotherapy regimens [1, 2], suggesting that not all AML patients can benefit from decitabine. As AML is a heterogeneous disease, the therapeutic effect of decitabine could be determined by many factors [3], and it is necessary to find suitable indicators for predicting the efficacy of decitabine to avoid overtreatment and optimize the treatment regimen. At present, research on molecular markers that can be used to predict the response to decitabine is relatively limited, and has mainly focused on the metabolic process of decitabine [4, 5]. Molecular markers that are associated with the mechanism underlying decitabine-mediated hypomethylation in the treatment of AML and can predict the response to the drug have not been reported.

Some studies have shown that hypomethylation in patients who achieved CR is more obvious than that in patients who did not achieve CR [6, 7]. Additionally, the response to hypomethylating drugs depends on the methylation density of CpG islands in specific gene [8], rather than the whole genome. Therefore, the methylation level of CpG islands in a specific gene is expected to be a valuable biomarker for predicting the efficacy of hypomethylation drugs. In addition to directly demethylating gene promoters, decitabine can also upregulate gene expression indirectly by interacting with upstream signaling pathways [9]. Thus, in AML patients receiving decitabine treatment, measuring only the methylation levels of a specific gene may not be sufficient to comprehensively reflect the response to decitabine.

As hypomethylation can upregulate the expression of tumor-suppressor genes [10], measuring the expression levels of genes regulated by hypomethylation is a more suitable strategy for evaluating the clinical response to decitabine. In this study, a combination of epigenetic and transcriptomic analysis was performed and a tumor-suppressor gene, BTG1, was identified to be involved in hypomethylation and the response to decitabine. BTG1 is widely involved in cellular processes such as cell division, DNA repair, transcriptional regulation and mRNA degradation, and inhibits cell proliferation and induces apoptosis [11]. Low expression of BTG1 in newly diagnosed AML was confirmed to be associated with CR and measurable residual disease (MRD) negativity after treatment with a decitabine-containing regimen.

The article "The predictive value of BTG1 for the response of newly diagnosed acute myeloid leukemia to decitabine" was retracted in 2024. Reasons: no approval from the institution; concerns about the data.

## Materials and methods

### Study design: patients and procedures

Bone marrow and peripheral samples were collected from newly diagnosed patients with de novo AML (not APL) enrolled in an open-label, randomized controlled clinical trial from September 2020 to April 2023. Among these patients, 54 were given decitabine + IA regimen, and 12 were given IA regimen; moreover, 8 healthy controls were collected. In this study, patients with newly diagnosed AML (not APL) were eligible if they met the following inclusion criteria: (i) patients aged 14–60 years, or aged 14–65 if the Eastern Cooperative Oncology Group (ECOG) score was < 2 points; (ii) patients with AML (not APL) who clearly met the WHO 2016 diagnostic criteria for AML; (iii) patients with newly diagnosed AML have not received chemotherapy; (v) patients with an ECOG score ≤ 2 points. The exclusion criteria were as follows: (i) a previous AML diagnosis; (ii) transformation of myelodysplastic syndrome (MDS) or other hematological diseases; (iii) central nervous system invasion; (iv) allergy to decitabine; and (v) heart dysfunction (ejection fraction < 50%), liver dysfunction (total bilirubin > 34 μmol/L), renal dysfunction (serum creatinine > 130 μmol/L), history of a fatal cerebrovascular events or severe infection. The decitabine + IA regimen was as follows: decitabine was administered initially (20 mg/m^2^/day, days 1–5), followed by idarubicin (10 mg/m^2^/day, days 4–6) and cytarabine (100–200 mg/m^2^/day, days 4–10). The IA regimen was as follows: idarubicin (10 mg/m^2^/day, days 1–3) and cytarabine (100–200 mg/m^2^/day, days 1–7). This study was approved by the medical ethics committee review board, and written informed consent was obtained from recipients in accordance with the Declaration of Helsinki before initiation of the study. This trial was registered with Chinese Clinical Trial Register (ChiCTR2000037928).

The initial response was evaluated according to NCCN guidelines, version 3.2023 [12] 21–28 days after completion of one treatment cycle, when complete hematologic recovery was achieved. The presence of MRD was evaluated according to the 2022 European LeukemiaNet (ELN) [13]. Bone marrow aspirates were used to assess the presence of MRD using multiparameter flow cytometry combined with real-time quantitative polymerase chain reaction (RT-qPCR) as follows.

(1) MRD assessed by multiparameter flow cytometry (MFC): CD45, CD34, CD117, CD13, CD33 and sideward scatter/forward scatter (SSC/FSC) were the core markers used to detect leukemia cells, with one or more of those markers CD7, CD11b, CD15, CD19, CD38, CD56, CD64 or HLA-DR abnormally expressed. MRD negativity was defined as < 0.1%. (2) For molecular MRD assessment: abnormal expression of genes associated with prognosis was evaluated by RT-qPCR. Expression of AML1-ETO, CBFβ-MYH11 and NPM1 < 0.01% was defined as MRD negativity [14, 15]. WT1 was used for molecular MRD assessment if no molecular marker was available at diagnosis, and MRD negativity was defined as WT1 expression < 0.6% [16]. Subjects were considered as MRD-negative when the MFC and molecular marker/WT1 expression data revealed MRD negativity in two consecutive samples.

The article "The predictive value of BTG1 for the response of newly diagnosed acute myeloid leukemia to decitabine" was retracted in 2024. Reasons: no approval from the institution; concerns about the data.

### Cell culture and drug treatment

Three human AML cell lines, Kasumi-1 (RRID: CVCL_0589), THP-1 (RRID: CVCL_0006), and MV4-11 (RRID: CVCL_0064), which were authenticated using short tandem repeat (STR) profiling within the last three years were purchased from the FuHeng Cell Center (Shanghai, China). Mycoplasma-free cells were cultured in RPMI-1640 medium supplemented with 10% (v/v) fetal bovine serum, 100 units/mL penicillin and 100 μg/mL streptomycin at 37 °C and 5% CO_2_. The Cell Counting Kit-8 (CCK-8) assay (Bioss, Beijing) was used to assess cell viability according to the manufacturer’s instructions. Cells were seeded into 24-well plates and treated with different concentrations of decitabine for 24 h, 48 h or 72 h. CCK8 (10 ul) was added to the culture medium and the cells were incubated for another 4 h. The absorbance of each well at 450 nm was measured using a microplate reader. The IC50 values of decitabine in the three cell lines were calculated according to the cell viability data. Apoptosis was evaluated using a FITC-Annexin V Apoptosis Detection Kit (BD Biosciences, Franklin Lakes, NJ, USA) following the manufacturer’s instructions.

### RNA-sequencing and data analysis

RNA was extracted from cells before and after decitabine treatment, and RNA-sequencing was performed using the Illumina HiSeq-PE150 platform. Differentially expressed genes (DEGs) between samples before and after decitabine treatment were filtered with according to the following criteria: *P* value < 0.05 and |log2FC(fold change)| (experimental vs. control) ≥ 0.8. Details about the sequencing coverage and quality statistics were shown in the Additional file 1. Transcriptome sequencing results of AML patients who achieved CR and those who did not achieve CR after standard “7 + 3” chemotherapy at initial diagnosis were downloaded from the public database gene expression omnibus (GEO) (http://www.ncbi.nlm.nih.gov/geo/). Based on the difference in their expression between samples from patients with CR and those with non-CR, DEGs were filtered, with the criteria of *P* value < 0.05 and |log2FC(fold change)|≤ 1. The significantly downregulated genes in samples from non-CR and significantly upregulated genes in samples from decitabine-treated cells were intersected.

The article "The predictive value of BTG1 for the response of newly diagnosed acute myeloid leukemia to decitabine" was retracted in 2024. Reasons: no approval from the institution; concerns about the data.

### Illumina infinium humanmethylation850k bead chip and data analysis

Methylation analysis of AML cell lines before and after decitabine treatment was performed using Illumina Infinium MethylationEPIC BeadChip (850 K Methylation EPIC arrays, a powerful tool for studying DNA methylation in tumors) (Illumina Inc, USA) [17]. DNA was isolated using the DNeasy Blood and Tissue Kit (Qiagen, Germany). The purity and concentration of DNA were estimated using Nanodrop 2000 spectrophotometer (ThermoScietific). Approximately, 500 ng of genomic DNA from each sample was subjected to sodium bisulfite conversion using the EZ DNA methylation Gold Kit (Zymo Research, USA) following the manufacturer’s standard protocol. Genome-wide DNA methylation levels were assessed using the 850 K Methylation EPIC arrays according to the manufacturer’s instructions. The array data were analyzed using ChAMP package in R to derive the methylation level. The methylation status of all the probes was calculated as the β value, which is the ratio of the methylated probe intensity to the overall probe intensity. CpG sites with |Δβ|≥ 0.20 (experimental vs. control) and adjusted *P* value ≤ 0.05 was considered as differentially methylated. The average β value of CpG islands were compared between decitabine treatment and control groups.

### Bisulfite sequencing PCR

Mononuclear cells were isolated from bone marrow or peripheral blood of AML patients with red blood cell lysate (Bioss, Beijing) followed by DNA extraction with DNeasy Blood & Tissue Kit (Qiagen). Bisulfite sequencing PCR (BSP) has been the gold standard for mapping DNA modifications including 5-methylcytosine for decades [18]. To ascertain which DNA sequence is responsible for regulating BTG1 transcription in AML cells, we searched the public database MEXPRESS [19] (https://mexpress.be/) and found that the methylation density of the CpG island cg08832851 in 3’untranslated region (UTR) of BTG1 was closely associated with BTG1 gene expression (r = − 0.503, *P* < 0.001) (Additional file 1: Fig. S1). Such methylation density on 3′UTR of BTG1 was determined using BSP [20] with EZ DNA Methylation-Direct™ Kit (Zymo Research, USA), and the primer targeting the 3′UTR of BTG1 was designed. The sequence on 3′UTR for designing primer was shown in Additional file 1: Fig. S2. The primer sequences used for BSP of BTG1 were shown in Additional file 1: Table S1. The BSP products were purified, cloned and inserted into into pMD19-T Vector (Takara, Tokyo, Japan), and transfected into DH5α competent cells (Vazyme Biotech Co., Piscataway). Five clones from each sample were sequenced (BGI Tech Solutions Co., Shanghai, China).

The article "The predictive value of BTG1 for the response of newly diagnosed acute myeloid leukemia to decitabine" was retracted in 2024. Reasons: no approval from the institution; concerns about the data.

### Real-time quantitative PCR (RT-qPCR)

The BTG1 mRNA expression levels of AML patients were analyzed by RT‑qPCR. Total RNA (10 μg per sample) was extracted from mononuclear cells isolated from AML patients and used to generate cDNA. The decitabine treated SKM-1 and THP-1 cells were collected for RNA extraction. cDNA was converted from 1 μg RNA using a reverse transcriptase kit (Vazyme, Nanjing). Gene expression was assessed using RT-qPCR following the instructions. Relative gene expression levels were analyzed using 2^−ΔΔCt^ method where Ct was the cycle threshold number normalized to GAPDH. Primers used for RT-qPCR were shown in Additional file 1: Table S1.

### Western blot

Cellular protein was isolated by lysis in RIPA buffer (Boster, Wuhan). Proteins in all samples were quantified with Bicinchoninic acid protein assay. Proteins of equal amounts from all samples were separated with SDS/PAGE gel (Bio-Rad, United States) and transferred onto PVDF membrane (Bio-Rad, United States). Bands were sealed with 5% skim milk, incubated in primary antibodies at 4 °C overnight, then in secondary antibodies at room temperature for 1 h, and then examined and analyzed using ChemiDoc™ XRS + with Image Lab™ Software (Bio-Rad, USA). BTG1 was tested using anti-BTG1 (ab151740, Abcam, British). β-actin was used as control (bs-0061R, Bioss, Beijing).

### Liposome-mediated BTG1 gene knockdown by transient transfection of small interfering (si) RNA

The sequences of siRNAs used for BTG1 knockdown and the negative control (NC) siRNA were shown in Additional file 1: Table S2. The siRNAs were transfected into Kasumi-1 and MV4-11 cells using LipoRNAi™ (Shanghai, China) according to the manufacturer’s instructions. After two days of culture, cells were used for further experiments, such as cell viability assay, Western blot and RT-qPCR.

### Statistical analysis

The expression differences of BTG1 between AML patients and healthy controls, and between AML cell lines before and after treatment with decitabine regimen were analyzed using t-test between two sets of data, or one-way ANOVA for comparisons among three or more sets of data. The correlation between methylation density and gene expression of BTG1, as well as the correlation between BTG1 expression in bone marrow and peripheral blood samples, was analyzed using Pearson’s correlation coefficients. The correlation between the methylation density and expression of BTG1 in three AML cell lines was analyzed by Spearman's rank correlation coefficient. The receiver operator characteristic (ROC) curve and Jordan index were used to analyze the maximum predictive value of BTG1 expression for the response to decitabine in AML patients at initial diagnosis. Continuous variables were expressed as the median and interquartile range (IQR) and were compared using independent t-tests for normally distributed data. Data were analyzed by the Mann–Whitney U-test when the data were not normally distributed. Categorical data were compared using the χ^2^ test, or Fisher's exact test when the data were limited. Analyses were performed with SPSS 25.0. *P* < 0.05 was considered as statistical significance.

The article "The predictive value of BTG1 for the response of newly diagnosed acute myeloid leukemia to decitabine" was retracted in 2024. Reasons: no approval from the institution; concerns about the data.

## Results

### Decitabine inhibits AML cell proliferation in vitro

The inhibitory effect of decitabine on the proliferation of AML cells was analyzed using CCK-8 assay and flow cytometry. As the decitabine concentration increased, the cell survival rate decreased and proliferation was inhibited (Fig. 1A). As the duration of decitabine prolonged, the cell survival rate decreased (Fig. 1B). The order of the AML cell lines in terms of the ability of decitabine to inhibit their proliferation was Kasumi-1 > THP-1 > MV4-11. Figure 1C showed the increased expression of Caspase-8 and Caspase-9, and decreased expression of BCL-2, as the concentration of decitabine increased. Figure 1D showed the apoptosis of AML cells treated with decitabine, with the order of the cell lines in terms of the apoptosis level was Kasumi-1 > THP-1 > MV4-11.

**Fig. 1:** Decitabine dose-dependently suppresses AML cell proliferation in vitro. **A** Viability of three cell lines after treatment with decitabine at different concentrations for 72 h. **B** Viability of three cell lines after treatment with 500 nM decitabine for different times. **C** Western blot analysis of cells treated with decitabine. **D** The cells apoptosis after treatment with decitabine (*P < 0.05 using ANOVA)

The IC50 of decitabine, the concentration of decitabine at which the proliferation of half of the cells were inhibited, in each cell line was calculated. The IC50 of decitabine was 250 nM in Kasumi-1, 500 nM in THP-1, and 1 μM MV4-11. Therefore, the order of these three AML cell lines in terms of the IC50 of decitabine was: Kasumi-1 < THP-1 < MV4-11. Decitabine was administered at a concentration of 500 nM for 72 h in subsequent experiments.

### The methylation and transcription analysis of AML cells treated with decitabine

850 K Methylation EPIC arrays were used to explore DNA methylation density before and after decitabine treatment in the three cell lines. A total of 210 overlapping genes with 308 overlapping methylation sites showed differentially decreased methylation after treatment with decitabine in all three cell lines (|Δβ|≥ 0.20 and *P* < 0.05) (Fig. 2A). Figure 2B showed decreased methylation sites after decitabine treatment in all three cell lines (|Δβ|≥ 0.20). Figure 2C showed differentially decreased methylation sites in each cell line (|Δβ|≥ 0.20 and *P* < 0.05). Kasumi-1 showed the mostly differentially decreased methylation after decitabine treatment, followed by THP-1 and MV4-11.

The article "The predictive value of BTG1 for the response of newly diagnosed acute myeloid leukemia to decitabine" was retracted in 2024. Reasons: no approval from the institution; concerns about the data.

**Fig. 2:** Comparison of the methylation density and gene expression in AML cells before and after treatment with decitabine. **A** Volcano plot of methylation changes before and after treatment with decitabine in all three cell lines. The green dots presented differentially decreased methylation sites while the black dots presented indistinctively decreased methylation sites. **B** Scatter plot of methylation changes in all three cell lines. The red dots presented decreased methylation sites (|Δβ|≥ 0.20) while the green dots presented decreased methylation sites (|Δβ|< 0.20). **C** Heatmap of differentially decreased methylation in each cell line. Different methylation sites were shown on the horizontal axis, with colors approaching red indicating high methylation density and blue indicating low methylation density. **D** Heatmap of upregulated genes (|log2FC|≥ 1); horizontal axis represented upregulated genes, with colors approaching red indicating high expression, and green indicating low expression. **E–G** Volcano plot of gene expression, with red dots indicating significant upregulation, green dots indicating significant downregulation, and blue dots indicating nonsignificant changes. **E** Kasumi-1 **F** THP-1 **G** MV4-11

RNA sequencing was used to analyze gene expression before and after decitabine treatment in the three cell lines. Figure 2D showed the upregulated genes with a |log2FC|≥ 1 in each cell line. Figure 2E–G showed the significantly upregulated genes and significantly downregulated genes (|log2FC|≥ 1 and *P* < 0.05). There were more upregulated genes than downregulated genes in Kasumi-1, the same number of, downregulated genes as upregulated genes in THP-1, and fewer upregulated genes than downregulated genes in MV4-11. The number of upregulated genes in the three types of cells was associated with the IC50 of decitabine.

### Combined analysis of experimental results and bioinformatics data

One of the important mechanisms by which decitabine inhibits leukemia cells is reversing the abnormal hypermethylation of tumor suppressor genes and upregulating their expression [21]. We know that if the expression of a weakly expressed tumor suppressor gene can be regulated by hypermethylation, it may be upregulated with decitabine. When newly diagnosed patients with a tumor suppressor gene did not achieve CR after treatment with the “7 + 3” regimen (cytarabine continuously for 7 days, and daunorubicin on each of the first 3 days), we hypothesized that such patients may respond to decitabine. Based on this hypothesis, genes meeting the two following criteria were selected.

1. Genes with low expression in newly diagnosed patients who did not achieved CR after treatment with the “7 + 3” regimen.
2. Genes upregulated after treatment with decitabine.

The article "The predictive value of BTG1 for the response of newly diagnosed acute myeloid leukemia to decitabine" was retracted in 2024. Reasons: no approval from the institution; concerns about the data.

Datasets GSE103424 [22] and GSE164894 [23] were downloaded from the GEO database, and detailed information was showed in Additional file 1: Table S3. DEGs at diagnosis between patients who achieved CR and those who did not achieve CR in the two datasets were compared. In GSE103424, the expression of 422 genes was significantly lower in patients with CR than those with non-CR. In GSE164894, the expression of 1004 genes was significantly lower in patients with CR than in those with non-CR.

Genes with low expression at diagnosis in patients who did not obtain CR in the datasets were intersected with genes upregulated by decitabine in the three cell lines using a Venn diagram (Fig. 3A), and four overlapping genes were identified: BTG1, CACNA2D2, MGAM, and TREM.

**Fig. 3:** Venn diagram and changes of the four overlapping genes in three cell lines treated with decitabine (IC50 of decitabine: Kasumi-1 < THP-1 < MV4-11). **A** Venn diagram. **B** The methylation density (β) of the 4 genes before treatment. **C** The changes of methylation density (Δβ) of the 4 genes after treatment with decitabine. **D** The mRNA (FPKM) of the 4 genes before treatment. **E** The changes of mRNA (log2FC) of the 4 genes after treatment with decitabine

### BTG1 is associated with the efficacy of decitabine in vitro

Subsequently, the methylation density (β values) and gene expression levels of the four overlapping genes in three cell lines before and after treatment with decitabine were analyzed to determine whether they were related to the IC50 of decitabine. The genes whose methylation density and expression level were most closely related to the IC50 of decitabine was selected.

1. The change in methylation density of BTG1 in three cell lines was significantly negatively correlated with the IC50 of decitabine (r = − 0.843, *P* = 0.004) (Fig. 3B).
2. The degree to which BTG1 was hypomethylated in three cell lines was significantly positively correlated with the IC50 of decitabine (r = 0.949, *P* < 0.001) (Fig. 3C).
3. The change in gene expression of BTG1 in three cell lines was significantly positively correlated with the IC50 of decitabine (r = 0.949, *P* < 0.001) (Fig. 3D).
4. The degree to which BTG1 was upregulated in three cell lines was negatively correlated with the IC50 of decitabine (r = − 0.474, *P* = 0.197) (Fig. 3E).

The article "The predictive value of BTG1 for the response of newly diagnosed acute myeloid leukemia to decitabine" was retracted in 2024. Reasons: no approval from the institution; concerns about the data.

According to findings (1), (2), and (3) mentioned above, BTG1-related changes in the three cell lines were significantly associated with the IC50 of decitabine. However, regarding CACNA2D2, only the change in the methylation density and the degree to which the gene was upregulated were significantly correlated with the IC50 of decitabine. Moreover, only the changes in the methylation density and gene expression of TREM1 were significantly correlated with the IC50 of decitabine, and no MGAM-related changes were significantly correlated with the IC50 of decitabine. Due to the most strong association with the IC50 of decitabine, BTG1 was selected for further analysis.

### Hypomethylation and upregulation of BTG1 after decitabine combined with IA treatment

Bone marrow and peripheral samples from 54 patients receiving decitabine + IA regimen, 12 patients receiving IA regimen, and 8 healthy controls were collected. The methylation density of BTG1 was measured using BSP and the primer targeting the 3′UTR of BTG1 was designed as described in the methods. As showed in Fig. 4, the methylation density of BTG1 was decreased from 60.0% to 0% in decitabine + IA treatment (Fig. 4A), whereas in IA treatment, it increased from 56.0% to 88.0% (Fig. 4B). When administered decitabine + IA regimen, the methylation density of BTG1 decreased from 100.0% to 16.0% in patient with CR (Fig. 4C), and decreased from 64.0% to 32.0% in patient with non-CR (Fig. 4D). The degree to which the methylation density of BTG1 decreased in patient with CR (84%) was higher than in patient with non-CR (32%).

**Fig. 4:** The methylation density of 3′UTR and gene expression of BTG1 in AML patients. **A** The methylation density of BTG1 was decreased in patients receiving decitabine + IA regimen. **B** The methylation density of BTG1 was increased in patients receiving IA regimen. The change of methylation density in patients with CR (**C**) and in patients with non-CR (**D)** in treatment with decitabine + IA regimen (the black beads presented methylated sites, the white beads presented unmethylated sites). **E** The change of BTG1 expression in patients receiving decitabine + IA regimen. **F** The change of BTG1 expression in patients receiving IA regimen. The change of BTG1 expression in patients with CR (**G**) and in patients with non-CR (**H)** in treatment with decitabine + IA regimen. **I** The negative association of the methylation density and gene expression of BTG1. **J** The association between BTG1 expression in bone marrow and that in peripheral blood samples

The mRNA expression levels of BTG1 in AML patients were detected using RT-qPCR. The mRNA of BTG1 in patients who received decitabine + IA regimen was significantly increased (*P* = 0.010) (Fig. 4E). In contrast, the mRNA expression of BTG1 in patients who received IA regimen was not significantly increased (*P* = 0.325) (Fig. 4F). Upon treatment with decitabine + IA regimen, the expression of BTG1 was significantly increased in patients who achieved CR (*P* = 0.004) (Fig. 4G) but not in patients who achieved non-CR (*P* = 0.962) (Fig. 4H). Thus, upregulation of BTG1 was more apparent in patients receiving decitabine + IA regimen than in patients receiving IA regimen, and was more apparent in patients with CR than in those with non-CR.

The article "The predictive value of BTG1 for the response of newly diagnosed acute myeloid leukemia to decitabine" was retracted in 2024. Reasons: no approval from the institution; concerns about the data.

Figure 4I showed the close negative association of the methylation density and gene expression of BTG1 (r = − 0.670, *P* = 0.002), suggesting that the methylation density on 3′UTR of BTG1 may regulate its expression of the gene. The association between expression and promoter methylation of BTG1 was also analyzed and found no significance correlation (Additional file 1: Fig. S3). Figure 4J showed the strong association of BTG1 expression between bone marrow and peripheral blood samples (r = 0.904, *P* = 0.035).

### Low BTG1 expression predicted response to decitabine + IA chemotherapy

In 54 newly diagnosed AML patients who received decitabine + IA regimen, the mRNA expression level of BTG1 was analyzed by RT-qPCR. The expression of BTG1 in AML patients was lower than that in healthy controls, and the expression of BTG1 in treated patients was higher than that in untreated patients (Fig. 5A). BTG1 expression at diagnosis in patients with CR was lower than that with non-CR, and BTG1 expression at diagnosis in patients with MRD negativity was lower than that in patients with MRD positivity (Fig. 5B).

**Fig. 5:** The association of BTG1 expression at diagnosis and efficacy of decitabine + IA regimen. **A** Comparison of BTG1 expression among healthy controls, untreated patients and treated patients. **B** Comparison of BTG1 in patients with CR and non-CR, and among patients with MRD negativity and MRD positivity. **C** ROC curve of BTG1 mRNA for predicting CR in training cohort. **D** ROC curve of BTG1 mRNA for predicting MRD negativity in training cohort. **E** ROC curve of BTG1 mRNA for predicting CR in variation cohort. **F** ROC curve of BTG1 mRNA for predicting MRD negativity in variation cohort. **G** Comparison of RFS in patients with high and low BTG1 expression. **H** Comparison of OS in patients with high and low BTG1 expression

These 54 newly diagnosed patients were divided into a training cohort (36 cases) and a variation cohort (18 cases), and the clinical characteristics of the two cohorts were compared in Additional file 1: Table S4. In training cohort, the predictive value of BTG1 to predict CR could be assigned with a sensitivity of 83.9% and a specificity of 80.0% when the BTG1 expression was < 0.318 at diagnosis, the area under the curve (AUC) = 0.868,* P* = 0.009 (Fig. 5C). The predictive value of BTG1 to predict MRD negativity could be assigned with a sensitivity of 87.5% and a specificity of 75.0% when BTG1 expression was < 0.229 at diagnosis, AUC = 0.826, *P* = 0.002 (Fig. 5D). In variation cohort, the predictive value of BTG1 to predict CR could be assigned with a sensitivity of 86.7% and a specificity of 100.0% when the BTG1 expression was < 0.292 at diagnosis, the AUC = 0.933,* P* = 0.021 (Fig. 5E). The predictive value of BTG1 to predict MRD negativity was assigned with a sensitivity of 100.0% and a specificity of 80.0% when BTG1 expression was < 0.292 at diagnosis, AUC = 0.892, *P* = 0.012 (Fig. 5F). Low expression of BTG1 could predict CR and MRD negativity in newly diagnosed AML patients who received decitabine + IA regimen.

The article "The predictive value of BTG1 for the response of newly diagnosed acute myeloid leukemia to decitabine" was retracted in 2024. Reasons: no approval from the institution; concerns about the data.

Subsequently, 54 newly diagnosed AML patients were divided into high and low expression groups according to BTG1 expression, with 0.292 as the cutoff (Additional file 1: Table S5). Patients with low BTG1 expression exhibited higher CR rate (97.5% vs. 50.0%, *P* < 0.001) and MRD negativity (85.0% vs. 14.3%, *P* < 0.001) than patients with high BTG1 expression. No difference was observed in 2-year RFS (86.4% vs. 57.8%, *P* = 0.436) (Fig. 5G) or 2-year OS (86.8% vs. 74.2%, *P* = 0.513) (Fig. 5H) between the two groups.

### Downregulation of BTG1 attenuated the inhibitory effect of decitabine

In order to investigate whether BTG1 is involved in the inhibitory effect of decitabine, siRNA was used to downregulate the expression of BTG1. Figure 6A showed that the mRNA of BTG1 in Kasumi-1 was downregulated after transfection with siRNA-1, siRNA-2 and siRNA-3 compared with siRNA-NC (*P* = 0.016, *P* = 0.008 and *P* = 0.002 respectively). The mRNA of BTG1 in MV4-11 was downregulated after transfection with siRNA-1 (*P* = 0.029) but not siRNA-2 or siRNA-3 (*P* = 0.133 and *P* = 0.057 respectively).

**Fig. 6:** Downregulation of BTG1 weaken the inhibitory effect of decitabine on AML cell proliferation. **A** Downregulation of BTG1 mRNA after transfection with siRNA. **B** Downregulation of BTG1 protein after transfection with siRNA. **C** The inhibitory effect of decitabine on Kasumi-1 and MV4-11 proliferation was weakened after transfection with siRNA-1 (*P < 0.05, siRNA-1 vs. siRNA-NC)

Similar to the mRNA of BTG1, the protein of BTG1 in Kasumi-1 was downregulated after transfection with siRNA-1, siRNA-2 and siRNA-3 compared with siRNA-NC. The protein of BTG1 in MV4-11 was downregulated after transfection with siRNA-1. Upon transfection with the siRNA-2 or siRNA-3, the BTG1 was not downregulated (Fig. 6B). Thus, siRNA-1 was selected for further experiments.

The article "The predictive value of BTG1 for the response of newly diagnosed acute myeloid leukemia to decitabine" was retracted in 2024. Reasons: no approval from the institution; concerns about the data.

After transfection with siRNA-NC, as the decitabine concentration increased, the cell viability of Kasumi-1 and MV4-11 cells decreased; however, after transfection with siRNA-1, the inhibitory effect of decitabine on cell proliferation was weakened (Fig. 6C), indicating that the inhibitory effect of decitabine on cell proliferation may depend upon the expression of BTG1.

## Discussion

With the development of high-throughput sequencing technology, the application of multi-omics analysis of the epigenome combined with transcriptome represents an important technical basis for analyzing tumor heterogeneity [24] and identifying tumor related biological markers [25]. In this study, a combination of epigenomic and transcriptomic analysis was performed to study the relationship between DNA methylation and gene expression before and after decitabine treatment. BTG1 expression was found to be closely related to changes in DNA methylation density, and was confirmed to predict the efficacy of decitabine-containing regimen in AML patients. BTG1 is a promising marker for optimization of individualized treatment in AML.

BTG1 gene, which is located on chromosome 12 and consists of two exons, encodes the anti-proliferation factor 1. BTG1 belongs to the anti-proliferative protein family and is mainly expressed in pancreas, heart and hematopoietic tissues [26]. BTG1 has the highest expression in the G0/G1 phase of cell cycle. It blocks cells in the G1 phase through the ERK/MEK pathway, inhibits the cell cycle progression, and mediates DNA programmed cell death, inducing beclin-1-dependent autophagy [27]. In hematopoietic stem cells, BTG1 maintains the resting state of hematopoietic stem cells in G1 phase, and regulates cell differentiation by upstream HLX, FOXO3a and PAX5 genes [26].

BTG1 is considered a tumor suppressor gene in lymphoid tumors and solid tumors. In non-Hodgkin lymphoma, BTG1 inhibits the proliferation of tumor cells by interacting with CNOT7 and CNOT8, and downregulated BTG1 leads to transformation and proliferation of tumor cells [28]. BTG1 expression in breast cancer cells is significantly lower than that in normal breast epithelial cells [29]. Low BTG1 expression in endometrial cancer is significantly associated with shortened overall survival [30]. Downregulation of BTG1 has been found in AML [31], but the clinical significance of BTG1 in AML is very limited. Only one research reported that the expression of BTG1 was significantly upregulated in patients who achieved CR, but not in patients who did not achieve CR after induction chemotherapy [32]. This study found obvious upregulation of BTG1 in patients who achieved CR after receiving decitabine + IA regimen, but not in patients who did not achieve CR, which was consistent with the above report.

The article "The predictive value of BTG1 for the response of newly diagnosed acute myeloid leukemia to decitabine" was retracted in 2024. Reasons: no approval from the institution; concerns about the data.

What is the association between the downregulated expression and DNA methylation of BTG1? In solid tumors such as colon cancer [27] and breast cancer [29], gene promoter hypermethylation is one of the important mechanisms leading to gene expression silencing. However, methylated CpG sites throughout the genome are numerous and complex. Unlike in solid tumors, the hypermethylation of the 3′UTR on CEBPA could affect CEBPA transcription in AML [33]. This study found that the downregulation of BTG1 expression was closely associated with the hypermethylation of the 3′UTR of BTG1 rather than the promoter. After decitabine treatment, a decrease in BTG1 3′UTR methylation and an increase in BTG1 gene expression were found, indicating that hypermethylation of BTG1 3′UTR may regulate the BTG1 gene expression. The regulation of BTG1 gene expression by hypermethylation of BTG1 3′UTR may be related to the following factors: Methylation can prevent many proteins including transcription factors from recognizing and binding with DNA [34]. 3′UTR hypermethylation can affect RNA exon splicing and polyadenylation [35]. 3′UTR hypermethylation can regulate microRNA expression to indirectly interfere with gene expression [36].

The downregulation of BTG1 expression in tumor cells can be reversed by the hypomethylating drug decitabine [29]. In this study, the inhibitory effect of decitabine on cell proliferation was weakened after BTG1 downregulation, suggesting that the inhibitory effect of decitabine on AML may be partially attributed to the hypomethylation and upregulation of BTG1. In addition to 3'UTR hypomethylation, BTG1 can also be upregulated by the upstream transcription factor FOXO3a [32]. Because decitabine can upregulate the expression of FOXO3a by hypomethylating its promoter [37], decitabine may also indirectly upregulate BTG1 expression through the DNMT1-FOXO3a-BTG1 pathway. Thus, decitabine can reverse the decreased expression of BTG1 in AML cells and exert an anti-leukemia effect through BTG1.

There are some limitations in this study: we identified BTG1 through in vitro experiments, and then verified its predictive value in clinical samples. However, we did not perform in vivo experiments on the relationship between low expression of BTG1 and the efficacy of decitabine. We are working on constructing an AML mouse model to perform such in vivo studies. In addition to DNA methylation, BTG1 is also regulated by the upstream factor FOXO3a. However, the upstream and downstream signaling pathways that regulate BTG1 expression need to be further studied.

The article "The predictive value of BTG1 for the response of newly diagnosed acute myeloid leukemia to decitabine" was retracted in 2024. Reasons: no approval from the institution; concerns about the data.

## Conclusions

BTG1 gene was identified as a marker for predicting response in AML using a combination of epigenome and transcriptome analysis that studied the relationship between DNA methylation and gene expression before and after treatment with decitabine. BTG1 expression was found to be closely related to the changes of DNA methylation density, and was confirmed to predict the efficacy of decitabine-containing regimen in AML patients. Low expression of BTG1 in newly diagnosed AML treated with decitabine-containing regimen was associated with CR and MRD negativity, suggesting that BTG1 is a potential marker to predict the response to decitabine.

### Supplementary Information

**Additional file 1. RNA Sequencing Coverage and Quality Statistics, Tables S1-5 and Figures S1-3. Table S1.** Primers of BSP and RT-qPCR for BTG1. **Table S2.** siRNA sequence of BTG1. **Table S3.** Datasets information. **Table S4.** Clinical characteristics of AML patients detected with BTG1. **Table S5.** Comparison of clinical characteristics between low and high BTG1 expression. **Fig. S1** The close association of gene expression and methylation density in BTG1. **Fig. S2** The sequence on 3’UTR used for designing primer. **Fig. S3** The methylation density of promoter and gene expression of BTG1 in AML patients.

## Data Availability

The original data of RNA-seq and 850 K Methylation EPIC arrays are available in the gene expression omnibus (GEO) repository, under GSE246874 (https://www.ncbi.nlm.nih.gov/geo/query/acc.cgi?acc=GSE246874).

## Abbreviations

AML: Acute myeloid leukemia
AUC: Area under the curve
BSP: Bisulfite sequencing PCR
CCK-8: Cell counting kit-8
CR: Complete remission
GEO: Gene expression omnibus
IQR: Interquartile range
MRD: Measurable residual disease
NC: Negative control
OS: Overall survival
RFS: Relapse-free survival
ROC: Receiver operator characteristic
STR: Short tandem repeat
